This article has been retracted.

# Feature Extraction of Athlete's Post-Match Psychological and Emotional Changes Based on Deep Learning

**DOI:** 10.1155/2022/2995205

**Published:** 2022-06-21

**Authors:** Shuchang Zhang, Fengjun Shan

**Affiliations:** ^1^Sports Teaching and Research Department, Jilin Business and Technology College, Changchun 130507, Jilin, China; ^2^College of Physical, Zhoukou Normal University, Zhoukou, Henan, China

## Abstract

Athletes have had to deal with significant shifts in the way they think about psychology and emotion before and after attending a match in their respective fields. It has become increasingly difficult for players of any sport to overcome these differences due to massive technological advancements that aid in analyzing the difficulties of an athlete. The trainer can use the results of the analysis to help motivate and prepare the athletes for the upcoming competitions. The analysis in this study is based on information about the athletes who competed in the Tokyo Olympics. Deep learning models were used to evaluate the study. Image feature detection can be accomplished through the application of a machine learning technique known as deep learning. It employs a neural network, a computer system that mimics the human brain's multiple layers. One or more unique features can be extracted from each layer. A deep learning model called the behavior recognition algorithm is used for the research. The questionnaire from the dataset was used to generate the results of the analysis.

## 1. Introduction

Athletes are considered real-life heroes as they represent the country in the events they participate in. Each athlete will face physical and mental challenges to achieve their best in participating sports. Athletes are expected to be strong and fast in their learning and performance. The goal of a person or sport is to enhance player development [1]. In contemporary sports culture, we are preoccupied with team-associated, individual statistics, and victimization of ancient measurements in every sport. In individual sports, a player's performance immediately translates into an accruing chance of victory. Team sports have a value-added complexity that facilitates the interplay of numerous individuals on a winning team. Understanding how a player processes data aids in coaching, motivating, and designing activities that will most effectively develop the athlete as an individual and as a member of the team [2]. The convergence of this subjective information with the target facts regarding how the athlete's brain functions and measurements relating to mental talents is captivating. Athletes are guided by health programs on the physical and mental issues they may face [3]. Previously, wellness programs were solely focused on physical health, with neither the player nor the team focusing on the mental state aspects of the sport. Sports enterprises will maintain athletes' well-being and improve their performance by designing a preventative wellness program personalized for each player.

To enhance performance while lowering player risk, a better understanding of the individual's mental talents is required. The intellect influences every player's skills and abilities, as well as their health; nonetheless, it is largely unknown in the sports industry [4]. Artificial intelligence (AI) offers a novel approach to understanding human minds, but it remains a broad term that is widely misunderstood, rife with both potential and hype, fact and fantasy [5]. The only definition of AI is software package systems that perform intelligently despite not being explicitly programmed. These systems learn to recognize and categorize input patterns, make and act on probabilistic forecasts, as well as operate without explicit rules or supervision [6]. AI and deep learning will identify latent patterns in encephalograms known as biomarkers that change over time and are related to the player's performance [7]. These biomarkers may be prone to living and delivering on the specific goals of each player and team.

Through example learning, AI enables the automation of biomarker identification, i.e., locating higher order feature areas that connect to specific phenomena. Deep learning finds patterns through the use of artificial neural networks [8]. Once upon a time, the most elegant neural network in our brain was shaped in this way. They have numerous layers to adjust automatic feature extraction from data—something that machine learning cannot do—with each subsequent layer victimizing the output from the preceding layer as input [9]. Deep learning focused on processing large levels of complexity, shapes, and amounts of data [10]. It will comprehend, learn, forecast, and adjust independently over time. At the same time, AI and deep learning help enterprises enhance player performance while limiting player danger by providing more insights from 100% of performance and health data at a scale that only automation can provide [11]. In this study, the deep learning model is used to analyze the athlete's psychological and stress levels.

The contribution of the study are as follows:

- Focused on determining the psychological and stress levels using deep learning model.
- It is based on information about the athletes who competed in the Tokyo Olympics.
- Aimed at analyzing the behavior of the athletes using the behavior recognition algorithm.

## 2. Related Works

Mental strength is a set of psychological traits that are essential for peak performance. Athletes, coaches, and sports psychologists have long questioned mental toughness as one of the most essential psychological traits connected with athletic achievement. Many studies have been conducted over the last decade to investigate the role of mental toughness in sporting success [12,13]. Its conceptualization and measurement, however, are without consent. This study intends to comprehensively investigate some of the new definitions and conceptualizations, as well as promote mental health. This review addresses both descriptive and analytical approaches to the analysis of mental toughness, with an emphasis on the patterns of development of this construct's assessment [14]. Whereas these discussions center on general characteristics of mental toughness, many of the concerns are pertinent to academics and practitioners concerned with assessing psychological factors connected to sport and exercise, as well as other performance or results settings [15]. The individuals should practice some preperformance tactics in advance so that they can handle the circumstances before feelings take control. When individuals or teams seek to achieve the same goals, competition may bring out the best or the worst in athletes, and the psychological demands are quite high. When physical abilities are equal, the competitor with the stronger mental attitude, who can regulate their mind before and during competitions, wins. Many athletes, however, incorrectly believe that mental aspects of performance are intrinsic and unchangeable [16]. In reality, consistent mental training can have an impact on performance similar to physical training; getting into the appropriate mindset before competing is among the most important parts of top performance. According to the research on Olympians, the combination of mental and physical awareness was a significant feature that distinguished the highest performing athletes from their lower performing peers at the Olympics [17]. Only cognitive characteristics were statistically related to the final Olympic scores of the three measured preparation stages (mental, physical, and technical). As the industry is expected, athletes and coaches respond in a variety of ways, with some becoming more introverted and silent, others more aggressive than normal, and others often disappearing into the background. Athletes exhibit their emotional emotions immediately during a difficult scenario, and this has a negative impact on their performance if they fail to manage their stress. As a result, it is critical to have a strategy in place to deal with preperformance stress [18,19]. Emotions are an important element of sport and competition, but if athletes do not manage them before the game, they can take control and affect their performance. Psychological strategies and routine application through mental management will help athletes prepare for improved performance [20,21]. The athletic trainers identified athletes with different psychological difficulties, presumably as they were aware of these potential components of sports injuries and considered them vital to the rehabilitation process [22]. It is also promising that they seemed to understand how to correctly detect the presence or absence of psychological disorders in athletes [23]. Furthermore, athletic trainers were reasonably aware of their obligations and felt competent in executing a variety of psychological strategies with athletes throughout rehabilitation. However, when asked to select appropriate psychosocial tactics, teacher assistants hesitated. That could be explained by the theoretical nature of most sports psychology classes [24]. As a result, including hands-on experience in physical exercise instruction should be recommended to ensure that trainers can handle applied scenarios with athletes. Experienced players have better self-regulation abilities than rookie ones. These abilities are frequently linked to preperformance as well as performance conditions. In keeping with a recent report prepared on recovery as well as performance in sports, we propose that self-regulation abilities are equally important for postperformance difficulties (e.g., recovery), and these skills should be trained to facilitate healing [25]. The study is also aimed at evaluating recovery as a dynamic self-regulatory process comprised of self-monitoring (i.e. awareness), cognitive and emotional control, and self-mastery (i.e. initiation into behavior). This, ideally, will influence future rehabilitation research (for example, through journal papers) and experts in increasing athlete resiliency. There is no existing study related to this subject. This study has been conducted to examine the performance of post-emotional and psychological changes. This study focused on evaluating the post-psychological and emotional changes of athletes using a deep learning approach.

## 3. Proposed Work

The architecture of the proposed work is seen in Figure 1. After the match, most of the athletes preferred self-talk for analyzing their emotions, efficiency, and anxiety.

In this research work, information on nearly 11,000 competitors representing 47 sports and 743 teams competing in the Tokyo Olympics in 2021 (2020) is considered. This dataset includes information on the athletes, coaches, and teams who competed, as well as gender-specific entries. It includes their names, the countries they represent, the discipline they compete in, the gender of the athletes, and the identifiers of the coaches.

The experiment group obtained either a week 1 (*n* = 36) or a week 8 (*n* = 38) self-talk (ST) intervention, whereas the group receiving no ST training. Following the initial intervention, the regression analysis (competition anxiety, voluntary control abilities, self-efficacy, as well as coaches' work enhancement) was measured thrice. ST training resulted in lower somatic anxiety levels and a state of awareness self-confidence, soul, self-efficacy, and performance, as expected. In addition, long-term training outperformed short-term training. Its tailored ST therapies may aid in improving the psychological states as well as the performance of junior athletes.

After the elite athletes are shot, the athlete's hits the crossbar or the size of ST. As a result, the equation at the time *t* as according is given in equations (1) and (2)

(1) $$\begin{array}{c} S_{x}=S_{1}^{*}\cos\;\theta , \end{array}$$

(2) $$\begin{array}{c} S_{y}=S_{1}^{*}\cos\left(-kt\right). \end{array}$$

The gravitational field  *h*, is one of the following curve used to calculate the trajectory of a core is given in equation.

(3) $$\begin{array}{c} Y=X\;\tan\;\theta -X^{2}\frac{h}{2V_{1}^{2}\cos^{2}\;\theta }. \end{array}$$

Let *X*=*P*,  *Y*=*F* − *h* be the requirement which the lands in the athletes center is given in equations (4) and (5)

(4) $$\begin{array}{c} \tan\;\theta =\frac{V_{1}^{2}}{hP}\left[1\pm \sqrt{1-\frac{2h}{V_{1}}}\left(F-h+\frac{hP^{2}}{2V_{1}^{2}}\right)\right], \end{array}$$

(5) $$\begin{array}{c} 1-\frac{2h}{V_{1}^{2}}\left(F-h+\frac{hP^{2}}{2V_{1}}\right)\geq 0. \end{array}$$

It can be solved for *V*_1_ given in

(6) $$\begin{array}{c} V_{1}^{2}\geq h\left[F-h+\sqrt{P^{2}+{\left(F-h\right)}^{2}}\right]. \end{array}$$

 *V*_min_ is the function of the level of *h*, as may be shown. The following formula can be used to calculate the incidence angle as the elite athletes as represented.

(7) $$\begin{array}{c} \tan\;\psi =\tan\;\theta -\frac{2\left(F-h\right)}{P}. \end{array}$$

It is assumed that when the hand is received, the athlete backboard is not taken into account; however, the size of athletes is assumed to have a diameter of *b* as well as the diameter of  *G*, which is represented in equation:

(8) $$\begin{array}{c} \sin\;\psi >\frac{b}{G}. \end{array}$$

Whenever the elite athletes touch the frame, its center can deviate from the frame's origin, as well as the maximum forward distance Δ*x*, after which it will be as in the equation.

(9) $$\begin{array}{c} \Delta x=\frac{G}{2}-\frac{b}{2\;\sin\;\psi }. \end{array}$$

If set *Y*=*P* − *h*, the result will be as in the equation.

(10) $$\begin{array}{c} x^{2}\frac{h}{2V_{1}^{2}}-x\;\tan+F-h=0. \end{array}$$

If you ask for help with *θ* and make *X*=*P*, you will be able to do the following equation.

(11) $$\begin{array}{c} \frac{bx}{b\theta }|x=L=\frac{P\left(V_{1}^{2}-PL\;\tan\;\theta \right)}{hP-V_{1}^{2}\sin\;\theta \;\cos\;\theta }. \end{array}$$

Substitute Δ*x*/Δ*θ* for the derivatives on the left to have the linear indicators between the divergences of a shot angle as Δ*x* and Δ*θ* and is represented in the equation.

(12) $$\begin{array}{c} \Delta \theta =\frac{hP-V_{1}^{2}\sin\;\theta \;\cos\;\theta }{P\left(V_{1}^{2}-hP\;\tan\;\theta \right)}\Delta x. \end{array}$$

## 4. Results and Discussion

Athletes were known to be decisive and quick in their learning and achievement. A person's or sport's purpose is to improve player development. In today's sports culture, we are fascinated with the team and individual statistics, ancient measurements in all sports. Individual achievement in individual sports quickly leads to an increased possibility of victory. Organized sports have such a value-added complication that it allows multiple people on a winning team to interact. Understanding that a player receives data helps with coaching, encouraging, and developing activities that will most likely reveal the details of the athlete's individuality and team membership.  Figure 2 indicates individuals in both the intervention and control groups, completed the tests and analysis once more. After a week, half of a control group was tested, with the remaining half examined after 8 weeks. Finally, depending on the athletes' schedules, we did the third information valuation about 5–6 weeks later to see if the therapies had any long-term effects (time 3). Participants in the control group were tested at the same time as those in the experimental and control groups. Deep learning enables organizations to improve player performance while reducing player risk by offering greater insights with 100% of health and physical data at a level that only automation can provide. The deep learning method is used to assess an athlete's psychological problems in performing well in sports. Athletes are supposed to be strong but also quick in their learning and performance.

Table 1 represents substitute Δ*x* and Δ*y* for the derivatives on the left to have the linear indicators between the divergence of a shot angle *x* as well as *y*. Values in the table are considered for Week 1 and Week 8 as in the database for the test and control groups. The attributes considered for the evaluation is also tabulated. A person's or sport's purpose is to improve player development. In today's sports culture, we are fascinated with the team and individual statistics victimization of ancient measurements in all sports. Individual achievement in individual sports quickly leads to an increased possibility of victory. Team sports have a value-added complexity that allows multiple persons on a winning team to interact. Understanding how a player processes data assists in coaching, encouraging, and structuring activities that will most effectively develop the athlete as an individual and as a team member. The confluence of this subjective knowledge with objective facts about how the athlete's brain functions and measurements linked to mental abilities is enthralling.

A deeper understanding of both the individual's cognitive capacities is essential to improve performance while minimizing player risk. Every player's analysis of athlete's self-talk challenges for group interaction affect cognition determines their talents and abilities, along with their condition; nonetheless, it is mostly unknown within sports industry. Artificial intelligence (AI) offers a novel approach to comprehending human minds, but it remains a broad term that is widely misunderstood, replete with both promise and hype, fact and imagination. The only description of artificial intelligence is different software systems can perform effectively despite not being pattern recognition. In Figure 3, investigation of possible social demographic as well as sports-related alterations among the three-groups with multivariate analyses of different but also square tests have been used. To evaluate the relations between men as well as women, athletes within the predictor variable at the time, multiple and multivariate analyses using descriptive statistics were undertaken for the entire predictor variable.

Table 2 represents the results of self-talk challenging exercises performed among the athletes who are grouped into six groups.

Athlete trainers were aware of the requirements and felt competent in implementing a number of psychological tactics with athletes during rehabilitation. When asked to choose appropriate psychosocial tactics, teacher assistants paused, which could be explained by the theoretical nature of most sports psychology lectures. As a result, including hands-on experience in physical exercise training should be encouraged to ensure that trainers are prepared to manage applied scenarios with athletes. Experienced players are better at self-regulation than inexperienced players. These abilities are frequently associated with both preperformance and performance situations. In accordance with a recent article on recovery and performance in sports, we recommend that self-regulation abilities are similarly crucial for post-performance issues, and that these skills should be cultivated to promote healing. In Figure 4, the coaches were unaware of the group task, but they were aware of the athletes' presence. It's impossible to say whether this information affects a coach's relationships with individual athletes as a result of their presentation ratings. I mention having the athletes evaluated by a third party, we also recommend that deep learning and hormone indicators be used to assess an organization's overall performance.

The results of the analyzed data are represented in Table 3.

A deeper understanding of the individual's mental abilities is essential to improve performance while minimizing player risk. Despite the fact that intelligence affects every player's talents and abilities, as well as their health, it is mostly unknown in the sports sector. Artificial intelligence (AI) offers a novel approach to comprehending human minds, but it remains a broad term that is widely misunderstood, replete with both potential and hype, fact and imagination. The only definition of artificial intelligence is software package systems that perform intelligently despite not being explicitly programmed. These systems learn to recognize and categorize input patterns, develop and act on probabilistic forecasts, and operate in the absence of explicit rules or supervision. In Figure 5, we can observe the coaches were unaware of the group task, but they were aware of the athletes' presence. It's impossible to say whether this information is partial to coaches' relationships with individual athletes with a result and their presentation ratings. In mention that the athletes be evaluated by a third person. We also recommend deep learning that hormone indicators be used to assess an organization's overall performance.

Table 4 represents the results that are influenced by the strategic knowledge and execution based on the framework, strategies, and the final results obtained. For each content category, the values are tabulated for the positive and the negative opinions.

In Figure 6, we can see that the individuals in the intervention and the control group completed the tests and analysis after the intervention program was completed (Time 2). After 1 week, part of a control group was tested, as well as the other half was examined following 8 weeks. Finally, dependent on the athletes' schedules, we did provide the data assessed 5 to 6 weeks earlier to see if therapies had any long-term effects (Time 3). A participant in the control group was tested at the same time as those in the experimental and control group. Team sports have the added complexity of allowing numerous people on a winning team to interact with one another. Understanding how a player processes data aids in teaching, encouraging, and planning activities that will best develop the athlete as an individual and as a team member. The intersection of this subjective information with objective data about how the athlete's brain functions and metrics related to mental talents is fascinating.

The descriptive statistical analyses for all variables are presented in Table 5 (a) and (b). Differences between the experimental group and control group at times were investigated using multivariate as well as multivariate analyses of variance in the same way as gender differences were investigated. With one exception, there were no significant differences in the regression model among the control group as well as the short-term of the investigational and control groups and the long-term experimental group (self-talk). As a result, the premise that the participants were correctly randomized into three groups and also that the groups did not change in the regression model prior to the commencement of the investigation appears to be justified.

## 5. Conclusions

Athletes' psychological and emotional behavior have to be stable before and after participating in any athletic or sports event. However, maintaining stability is a challenge for all the athletes, rigorous training and encouragement can make the ends meet the thirst for success both in their career and personal. This study deployed a behavior recognition algorithm-based deep learning technique for evaluating the post-psychological characteristics of athletes. It also evaluates the mental health and emotional balance experienced by the athletes. The study results proved that the proposed model has provided an accuracy of 89%. For future research, it is highly recommended to determine the impact of deep learning toward pre -and post-psychological situations of athletes.

## Figures and Tables

**Figure 1:** Architecture of the proposed system.

**Figure 2:** Substitute Δ*x* and Δ*y* for the derivatives on the left to have the linear indicators between the divergences of a shot.

**Figure 3:** Analysis of athlete's self-talk challenges for the group interaction effect.

**Figure 4:** Analysis to investigate athlete's influenced strategy using deep learning method.

**Figure 5:** Analysis to investigate the athlete's influenced strategic framework.

**Figure 6:** Analysis of athletes to investigate the athletes influenced strategic analysis of covariance.

**Table 1:** Result of the linear indicators.

Group	Week	Excellent satisfied	Fulfillment	Not so pleased	Not pleased	Total
Text group	One	66	30	50	90	87
	Eight	80	35	7	0	100
Control group	One	42	48	20	0	85
	Eight	45	45.5	12.00	0	100

**Table 2:** Results of a self-talk challenge exercise.

Groups	Total match frequency	Collaboration times that are reasonable	Self-talk challenge (%)
Group 1	28	21	75
Test control (G1)	21	13	61
Group 2	26	17	65
Test control (G2)	19	11	60
Group 3	27	20	71
Test control (G3)	20	12	58

**Table 3:** Results of the analyzed data.

S.no	Investigate athlete's	Yes		General		No	
		DL method	Proportion	DL method	Proportion	DL method	Proportion
1	Is it of any use?	75	93.5	7	8.6	0	0
2	How can you boost your motivation to learn?	87	100	0	0	0	0
3	Is it possible to cultivate a desire to learn?	78	99.2	1	1.67	0	0
4	How can you master information faster?	79	95.86	5	6	0	0
5	How can you improve your analytical skills?	75	90	7	9.3	0	0

**Table 4:** Results are influenced by strategic knowledge as well as execution.

Content	Test control			
	Prior to attempting an experiment, yes	After test (yes)	Prior to attempting an experiment, no	After test (no)
Framework	37.8 ± 7.3	58.1 ± 8.2	37.3 ± 7.0	56.2 ± 7.1
Strategies	21.7 ± 24.3	66.2 ± 3.9	21.7 ± 5.2	31.9 ± 4.0
The end result	89.1 ± 25.4	161.2 ± 18	89.1 ± 26	153.5 ± 28.1

**Table 5:** (a, b): National anxiety, negative emotionality, voluntary control skills, self-talk efficacy, but also team manager performance mean score and standard deviance for three measurement points of time, as well as the results of 3 (Time) 3 (Group) multivariate and multivariate regression analysis of covariance for state anxiety, negative emotionality, voluntary control skills, self-efficacy, as well as coach-rated performance.

(a)											
Variable				(DL *V*) *F*-time		*P*; ѱ^2^		(DL V) *F T* × *G*		*P*; ѱ^2^	
National anxiety: WAL -S				1.89		0.15; 0.04		2.65		0.13; 0.36	
Somatic national anxiety				1.67		0.26; 0.03		2.87		0.16; 0.18	
Reasoning national anxiety				1.98		0.27; 0.03		1.43		0.28; 0.12	
National self-confidence				3.63		0.09; 0.05		3.65		0.02; 0.18	
Trait of anxiety: WAL-T				5.89		<0.001; 0.06		1.76		0.30; 0.13	
Trait anxiety of somatic				10.93		<0.001; 0.17		0.49		0.60; 0.12	
Disquiet				7.62		<0.001; 0.04		1.54		0.47; 0.13	
Meditation disruption				6.78		<0.001; 0.06		1.37		0.27; 0.14	
Volitional control skills (VCS)				1.45		0.23; 0.18		2.34		0.007; 0.30	
Self-talk optimization				2.78		0.007; 0.02		6.89		<0.001; 0.25	
Self-talk impediment				2.25		0.85; 0.05		1.57		0.18; 0.14	
Energy shortfall				1.89		0.97; 0.07		1.79		0.56; 0.15	
Loss of effort				2,367		0.08; 0.06		0.75		0.87; 0.12	
Self-talk efficacy				11.68		<0.001; 0.17		4.40		0.003; 0.20	
Coach performance				10.26		<0.001; 0.28		3.76		0.02; 0.28	

(b)											
Control group			Short-term intervention				Long-term intervention				
Time-1	Time-2	Time-3	Time-1	Time-2		Time-3	Time-1	Time-2		Time-3	
*V*_*c*_			*V*_STI_				*V*_LTI_				
*S*_*c*_			*S*_STI_				*S*_LTI_				

National anxiety: WAL-S											
5.93a 2.51	6.85b 2.78	6.34a 2.72	6.69a 2.52	5.96b 2.49		5.46c 1.67	7.22a 2.86	6.45b 1.98		6.46b 2.69	
7.40 2.87	7.84 3.00	8.01 3.55	8.07 2.67	7.30 2.69		8.13 3.74	8.68 3.21	7.39 2.82		7.64 3.01	
10.78a 2.89	12.19b 2.48	9.46a 2.59	9.95a 2.58	10.71a 3.28		10.38a 3.24	9.99a 2.45	10.86b 2.21		11.62c 2.97	
Trait of anxiety: WAL-T											
10.32 3.76	9.20 3.58	8.60 3.40	9.84 3.41	9.00 3.74		9.31 3.33	9.84 2.81	8.73 3.63		8.57 3.79	
10.04 3.13	9.58 2.97	9.08 3.46	9.19 2.95	8.37 3.70		8.82 3.43	9.99 3.38	8.57 3.22		8.32 3.42	
6.04 1.59	5.80 1.44	6.16 1.99	7.48 2.99	6.52 2.69		6.42 2.47	6.61 2.04	5.79 1.93		5.89 1.91	
Volitional control skills (VCS)											
58.98a 11.43	56.32b 12.53	56.68c 12.18	67.29a 19.23	60.56a 13.32		59.98a 13.63	55.68a 17.19	65.16b 12.43		65.47c 17.91	
10.80 3.87	11.80 4.60	12.52 4.74	13.87 5.61	12.61 5.89		13.13 5.33	12.88 4.48	12.27 5.01		12.58 4.13	
9.05 5.63	10.07 6.31	12.18 7.91	10.54 8.47	9.85 6.98		9.18 7.71	9.32 6.93	9.98 7.20		11.60 8.35	
8.08 3.44	8.08 5.50	8.96 6.33	10.52 6.39	9.47 6.67		9.41 5.78	9.28 5.34	7.80 5.49		8.37 5.87	
27.27a 3.84	37.78a 3.92	36.81a 4.33	22.09a 3.42	29.91b 4.86		29.25a 4.89	27.76a 5.73	37.12b 5.68		41.53b 5.46	
28.39a 5.81	21.97a 4.35	21.72a 5.34	23.49a 3.96	27.14a 4.86		28.30a 6.09	25.16a 4.32	38.32b 3.39		28.62b 4.71	

## Data Availability

The data used to support the findings of this study are included within the article.
